The article "Anatomical and Imaging Study on the Optimum Entry Point and Trajectory for Anterior Transpedicular Root Screw Placement into the Lower Cervical Spine" was published in 2022. Journal: Comput Math Methods Med.

# Anatomical and Imaging Study on the Optimum Entry Point and Trajectory for Anterior Transpedicular Root Screw Placement into the Lower Cervical Spine

**DOI:** 10.1155/2022/8159570

**Published:** 2022-08-09

**Authors:** Jihui Zhang, Liujun Zhao, Jingfei Xu, Yongjie Gu, Liang Yu

**Affiliations:** ^1^Department of Spinal Surgery, Ningbo No. 6 Hospital, Ningbo, 315040 Zhejiang Province, China; ^2^Department of Medical Insurance, Ningbo No. 6 Hospital, Ningbo, 315040 Zhejiang Province, China

## Abstract

**Objective:**

To study the optimum entry point and trajectory for anterior transpedicular root screw (ATPRS) placement into the lower cervical spine (LCS), so as to provide a basis for clinical application.

**Methods:**

A retrospective analysis of cervical CT images of patients who underwent cervical CT examination in the Spinal Surgery of Ningbo No. 6 Hospital from January 2020 to August 2021 was conducted. The data were obtained and modeled. On the coronal plane, the vertebral body (VB) between the anterior midline of cervical vertebral segments C_3-7_ and the left P line (by drawing the line parallel to the anterior midline of the VB at the intersection of the anterior edge of the Luschka's joint and the upper endplate) was equally divided into 9 zones (a-i). The ideal entry point and path of cervical ATPRS were designed and recorded. Additionally, 7 cadaveric specimens were selected, and the screw placement parameters were regenerated according to the above methods for screw placement.

**Results:**

Zone i of each segment, with the longest screw length, was the best area for screw placement. In all patients, the horizontal angles of vertebrae C_3-7_ in zones a, d, and g, zones b, e, and h, and zones c, f, and i showed a gradually decreasing trend. The sagittal angle range of C_3-7_ in all patients showed a gradually increasing trend in zones a-c, d-f, and g-i. The distance from the anterior midline of C_3-7_ to the P line increased in all patients, and the distance was longer in males than in females, with statistical significance. Pedicle screws were successfully inserted in all the 7 cadaveric specimens.

**Conclusions:**

ATPRS placement can be used for LCS internal fixation, and the precise screw placement parameters can be simulated by the software, which provides theoretical basis for its future clinical application.

## 1. Introduction

The change of lifestyle in modern society has driven the continuously rising incidence of cervical spine injury (CSI), with degenerative diseases, trauma, and infection of the lower cervical spine (LCS) frequently occurring in the anterior column of the vertebral body (VB) [1, 2]. Clinically, surgical treatment is mainly adopted to relieve spinal cord and nerve root compression, restore the normal sequence and physiological curvature of cervical spine (CS), and rebuild the stability of CS. Anterior cervical decompression and fusion is a common method to treat lower cervical diseases [3, 4], most of which are fixed with unicortical cervical vertebral screws, with a good fixation effect for patients with single-level cervical diseases. However, a combination of anterior and posterior surgery is usually required for those with single-level three-column injury or multilevel anterior compression treated by anterior vertebral screws, with anterior surgery for decompression and posterior surgery for fixation. However, the biomechanical stability of traditional anterior cervical plate and screw fixation is not satisfactory [5, 6]. Although posterior pedicle screws or lateral mass screws can provide sufficient stability for patients with multilevel internal fixation, this procedure undoubtedly lengthens the operative time of patients and increases surgical trauma, complications, and costs [7–9].

The article "Anatomical and Imaging Study on the Optimum Entry Point and Trajectory for Anterior Transpedicular Root Screw Placement into the Lower Cervical Spine" was published in 2022. Journal: Comput Math Methods Med.

There are two anterior cervical internal fixation methods: vertebral screws, which are widely used in clinical practice, and pedicle screws, which are limited by difficulty in screw placement [10, 11]. Therefore, how to achieve the dual purpose of decompression and fixation at the same time in LCS surgery through anterior approach has become a research hotspot in recent years. As an alternative, the anterior transpedicular screw (ATPS) technique, applied clinically by Aramomi et al. [12], has gradually been extensively used for cervical stabilization due to the combination of the advantages of anterior approach with superior biomechanical properties of cervical pedicle fixation [10, 13, 14]. In general, pedicle fixation is considered risky because of the anatomical relationship of the cervical pedicle, which is close to important structures such as vertebral arteries, spinal cord, and nerve roots [15, 16].

Therefore, precise screw insertion is the key to successful clinical application of ATPS. Under this circumstance, we proposed a novel anterior screw technique called anterior transpedicular root screws (ATPRSs) for anterior cervical arch foundation, which is also the novelty of this study. At the same time, due to ethnic anatomical differences, there are limited anatomical and imaging studies related to this technique in China. Thus, the motivation of this paper is to study and measure the applied anatomy and CT of the lower cervical vertebra from the anterior approach, in order to provide anatomical and imaging-related parameters for ATPRS implantation in the LCS.

The article "Anatomical and Imaging Study on the Optimum Entry Point and Trajectory for Anterior Transpedicular Root Screw Placement into the Lower Cervical Spine" was published in 2022. Journal: Comput Math Methods Med.

## 2. Data and Methods

### 2.1. General Information of Samples Collected In Vivo

Cervical CT images of patients undergoing cervical CT examination in the Spinal Surgery of Ningbo No. 6 Hospital from January 2020 to August 2021 were collected. Inclusion criteria: Adult patients who visited Spinal Surgery and underwent cervical CT examination, with no obvious LCS deformity or history of cervical surgery (to eliminate the measurement error caused by the interference of surgery or internal fixation), and complete imaging data were enrolled. Exclusion criteria: Patients with fracture, deformity, tumor, and obvious degeneration or previous cervical surgery history were excluded, as well as those aged under 25 or over 70. According to the inclusion and exclusion criteria, 39 patients were finally enrolled, including 22 males and 17 females, with an age range of 28-66 years (mean: 39.3 ± 8.9). This study was approved by the hospital Ethics Committee (Ethics Number: NBU-2021-021). Because of the retrospective nature of this study, the requirement for informed consent was waived.

### 2.2. Model Reconstruction

The original CS CT data of 39 patients in Dicom format were imported into the Mimic 17.0 software (Mimics 17.0, Materialize, Belgium) for analysis. After reading CT sequence images, the threshold value of CS was selected to obtain the original mask. Then, three-dimensional (3D) reconstruction was performed to establish 3D images of vertebrae C_3-7_ successively through multilayer mask processing. After smoothing and triangular patch (TriPatch) trimming, the complete 3D images of vertebrae C_3-7_ were obtained and saved.

### 2.3. Virtual Screw Placement and Data Measurement

In order to avoid measurement biases caused by subjective factors of the gauger, all the following data were repeatedly measured by two researchers skilled in the operation of mimics software, and the measured data results were averaged as the final data.

The retrieved 3D images of C_3-7_ levels were displayed with the highest transparency to establish contour lines. On the coronal plane, a line parallel to the anterior midline of the VB at the intersection of the anterior edge of the Luschka's joint (uncovertebral joint, UVJ) and the superior endplate was made, which is called the P line, and the VB between the anterior midline of the C_3-7_ levels to the left P line was evenly divided into 9 zones (a-i), by referring to our previous study [17]. Then, a cylinder with a diameter of 3.5 mm was drawn by MEDcad module instead of screws for simulation of screw placement. Pedicle screw placement: After transparentizing the 3D reconstruction of the VB, the posterior wall of the VB was used as a reference to make it perpendicular to the screen, with the overlap of the upper and lower edges of the posterior wall of the VB and no lateral inclination as the standard. Then, the VB was restrained. The transverse distance of the vertebral canal was used to locate the central line of the VB, and the horizontal vertical line perpendicular to the central line was established by the anterior edge of the VB. The VB was then rotated to show its sagittal view. Then, the posterior wall of the VB was made perpendicular to the lower edge of the screen, and the projection line of the posterior wall was overlapped and constrained again to make a vertical line perpendicular to the center line. The horizontal, coronal, and sagittal planes of the VB were determined by the principle of two lines determining one side through the center line, the horizontal vertical line, and the vertical line. In the viewing window, the VB was set to a horizontal plane in which the VB was rotated so that the pedicle was perpendicular to the lower edge of the screen to facilitate screw placement. The cylinder was moved slowly to ensure that it was embedded in the vertebra. Fine-tuning was performed in sagittal, coronal, and horizontal windows to make the simulated screw placement in the best position. That is, the head of the screw was located at the intersection of the posterolateral edge of the VB and the axis of the pedicle on the horizontal plane and at the lower edge of the pedicle on the sagittal position. The caudal end of the screw was located at the center point of 9 zones equally divided between the midline of the anterior edge of VB and the left P line. The method of bilateral screw implantation was consistent.

The article "Anatomical and Imaging Study on the Optimum Entry Point and Trajectory for Anterior Transpedicular Root Screw Placement into the Lower Cervical Spine" was published in 2022. Journal: Comput Math Methods Med.

Through the measurement module of the Mimics software, the measurement file was established to determine the position and length of the screw. The horizontal plane angle (*α*), sagittal plane angle (*β*) of the anterior pedicle screw, and the distance from the midline of anterior edge of VB to the P line were measured. Related data of each VB was recorded using the Excel software.

### 2.4. Nailing of Cadaveric Specimens

Seven adult cervical vertebra specimens treated with formaldehyde were selected, including 4 males and 3 females aged from 29 to 58 years (mean: 43.7 ± 10.1). After eliminating bone defects, deformities, and obvious degeneration by CT examination, the soft tissue in front of the cervical VB was gradually and thoroughly removed, the prevertebral fascia was incised, and the VB was exposed, with the strip width to the bilateral UVJs. The prepared specimens were refrigerated at -20°C and taken out 24 hours before the formal experiment.

Seven CS specimens were randomly numbered and scanned by CT, and the related parameters were measured by the Mimics software in the same way as adult CS CT images. After thawing the specimen at room temperature and fully exposing the VB and other bone structures, the screws were gradually inserted under the guidance of C-arm X-ray machine and Kirschner wires, and ATPRS were placed under X-ray fluoroscopy. Subsequently, the screw trajectory was observed to determine whether the screw was located in the bone. After confirming that the upper wall of the channel and the left and right lateral walls were not damaged, the safety of screw placement was reconfirmed by anteroposterial-lateral fluoroscopy. Following screw placement, a CT scan was performed to determine the position of the screw and whether the screw was inserted safe and effective. Also, the specimen was dissected along the screw with a pendulum saw to check whether the screw penetrated the bone surface or damaged the surrounding structure, and the screw trajectory was observed.

The article "Anatomical and Imaging Study on the Optimum Entry Point and Trajectory for Anterior Transpedicular Root Screw Placement into the Lower Cervical Spine" was published in 2022. Journal: Comput Math Methods Med.

### 2.5. Statistical Processing

Statistical analysis was made by SPSS 22.0 (IBM, NY, USA). Mean ± SD was used to indicate the measurement data of normal distribution, and an independent samples *t*-test was performed. For the intragroup comparison of screw placement zones, a paired sample *t*-test was used. A significance level of two-tailed *α* = 0.05 was used in all analyses.

## 3. Results

### 3.1. Screw Lengths in Each Zone of Cervical Levels C_3-7_

After software simulation of screw placement, it was found that the APSs could be placed at the cervical levels C_3-7_ in all patients. The optimal areas were screw lengths over 22 mm for males and 20 mm for females, as shown in Table 1.

### 3.2. Horizontal Angles of APSs in Each Zone of Cervical Levels C_3-7_

The screw horizontal angles of all patients are shown in Table 2. The horizontal angle differed significantly between males and females at different cervical levels (*P* < 0.05). However, no significant difference was present in angles between zones a, d, and g of C_3-7_ segments in all patients (*P* > 0.05). Nor was there any obvious difference in the horizontal angle between zones b, e, and h and zones c, f, and i (*P* > 0.05), all of which showed a decreasing trend in the angle.

### 3.3. Sagittal Plane Angles of APSs in Each Region of Cervical Levels C_3-7_

The sagittal angle showed significant differences between male and female at different cervical levels (*P* < 0.05). However, there was no significant difference in the angle between zones a, b, and c of C_3-7_ segments in all patients (*P* > 0.05). Also, zones d, e, and f were not evidently different from zones g, h, and i in the sagittal angle (*P* > 0.05), all of which showed an increasing trend (see Table 3).

The article "Anatomical and Imaging Study on the Optimum Entry Point and Trajectory for Anterior Transpedicular Root Screw Placement into the Lower Cervical Spine" was published in 2022. Journal: Comput Math Methods Med.

### 3.4. Distance from Midline of Anterior Edge to P Line at Cervical Vertebra C_3-7_

As shown in Table 4, from C_3_ to C_7_, the distance from the anterior midline of the VB to the P line increased gradually, with that of C7 being the longest and a distance shorter in females than in males (*P* < 0.05). Subsequently, screw placement was carried out on cadaveric specimens according to simulated nail placement parameters, which proved the feasibility of nail placement, as shown in Figure 1.

## 4. Discussion

At present, anterior CS plate fixation is widely used, in which 13-15 mm vertebral mono- or bicortical screws are mostly used as the fixation screws, with better fixation strength for patients undergoing single-level surgery [18]. However, for senile osteoporosis patients and those with cervical multilevel decompression, this procedure can easily lead to loosening of internal fixation. Currently, there is no relatively stable and reliable fixation method in clinical practice [19]. Biomechanical studies have shown that the pedicle is the toughest part of the vertebrae, and its cortical bone is cylindrical with a small amount of cancellous bone in the middle. This structure has a good holding force on screws, and the stability provided by pedicle screw fixation is obviously better than that provided by anterior cervical locking plate system, posterior spinous process wire fixation, and transarticular plate/screw fixation [19–22]. Due to the special anatomical characteristics of the pedicle of the LCS, any deviation during the operation will cause serious consequences. If the screw path is too high, it is easy to damage the nerve root, while too internal a screw path is prone to spinal cord injury; if the screw path is too lateral, it can easily damage the vertebral artery [23]. As the application of anterior cervical pedicle screw internal fixation technology is still in its initial stage, there have been no reports of injury of arterial spinal cord and nerve roots or failure of internal fixation. Similar to posterior cervical pedicle screw fixation, anterior pedicle screw fixation has the risk of complications such as damage to vertebral artery spinal cord and nerve roots, as well as complications such as hoarseness, esophageal injury, cerebrospinal fluid leakage, and internal fixation failure caused by traditional anterior surgery [24, 25]. At the same time, most scholars believe that successful pedicle screw placement depends on three factors [26], namely, the location of the entry point, the appropriate placement angle in the transverse and sagittal planes, and the appropriate screw diameter and length. Hence, precise measurement of parameters related to these elements becomes the key to ensuring surgical success.

The article "Anatomical and Imaging Study on the Optimum Entry Point and Trajectory for Anterior Transpedicular Root Screw Placement into the Lower Cervical Spine" was published in 2022. Journal: Comput Math Methods Med.

In this study, the Mimics software is used to carry out 3D reconstruction with CT images to realize simulation operation and 3D measurement. The simulation of screw placement can be repeated in the software, which is helpful to the study of the best entry area and trajectory of screw placement. The basic research of anterior pedicle screw placement using the Mimics software involves the question of reliability in comparison with the real thing. The samples included in the research were 3D models reconstructed by CT scanning. Although there is a certain difference between the surface treatment and the real object, there is no distortion in the angle; moreover, this technology is a CT scan orientation, so the distribution of the spatial structure of the model is consistent with the real object. At present, a large number of studies have used the Mimics software to build cervical VB for finite element analysis and clinical surgical procedures [27–29]. In this study, the screw placement area was refined and divided into 9 zones, and the screw placement parameters of each zone were analyzed. The results indicated that screws larger than 22 mm could be placed in men and more than 20 mm in women. Zone i was the optimal entry point among all the 9 zones, with the longest screw length. The screw diameter, however, is mainly determined by the pedicle width. Generally, the screw diameter should be smaller than the pedicle width of the corresponding segment and larger than the relatively small cancellous bone core, so that the thread can be cut into the cortical bone, thus maximizing the pull-out force and bending strength. In this study, the screw placement was set to 3.5 mm and its feasibility was demonstrated. The pedicle screw diameter can therefore be selected as a baseline safe value of 3.5 mm and adjusted as appropriate. This study also found no statistical significance in the horizontal angle of C_3-7_ on the same sagittal plane. But the horizontal angle of different sagittal planes showed statistically significant differences with a gradually decreasing trend, among which the angles of zones a, d, and g were the largest. Therefore, when nailing in these areas, the inclination angle should be the largest. The sagittal angle at the same level had no statistically significant difference, but the sagittal angle at different levels showed a statistically significant difference with a gradually increasing trend, which is similar to our previous findings [30]. The method used here was first proposed in our previous research [17] and was first applied on cadaveric specimens in this study. Before surgery, the CT data of patients was imported into the software, and the screw placement was simulated in the optimal area to determine the final entry area and trajectory. It was also observed in this study that the distance from the midline of the anterior edge of C_3-7_ to the anterior edge of the UVJ gradually increased. Finally, we further applied this method to cadaveric specimens and confirmed its feasibility. However, this study mainly used fluoroscopy-guided free-hand screw placement, and despite successful placement in cadaveric specimens, the study demonstrated a 21.7% incidence of critical pedicle rupture in the axial plane [13]. Patton et al. [11] found that catastrophic screw placement occurred in 33.3% of the patients with fluoroscopy-guided free-hand screw placement, compared with a significantly lower but still high incidence of 16.7% in the image-guided group. It is shown that patient-specific drill templates (PDTs) made by three-dimensional printing technology (3DP) had favorable effectiveness and accuracy in assisting cervical transpedicular screw placement [31, 32].

The article "Anatomical and Imaging Study on the Optimum Entry Point and Trajectory for Anterior Transpedicular Root Screw Placement into the Lower Cervical Spine" was published in 2022. Journal: Comput Math Methods Med.

This study still shows room for improvement. First of all, the data collected are all from CT reconstruction images, which inevitably leads to human errors. Besides, in the actual clinical operation, it is relatively difficult to find the optimum entry point in clinical screw placement because most patients requiring surgery had CS degeneration of varying degrees. And in view of the accuracy of this screw placement method, it is necessary to strictly study and analyze the patients with surgical indications. Moreover, the sample size of this study is small, so it is necessary to further study the biomechanical stability and accuracy of this screw placement method. In a word, ATPRS placement into the LCS is a feasible internal fixation technique, but its clinical application value needs further systematic analysis and research.

## 5. Conclusion

In summary, anatomical and radiographic measurements demonstrate that ATPRS can be used as a means of internal fixation of the lower CS in clinical practice. Due to the accuracy of this operation, it should not be used as a routine operation, and patients with surgical indications should be strictly selected. But we think that as research continues and technology advances, ATPRS will be further promoted and applied.

## Figures and Tables

**Figure 1:** Screw placement in cadaveric specimens.

**Table 1:** Comparison of screw lengths in different levels and zones of cervical vertebrae (cm).

	C_3_		C_4_		C_5_		C_6_		C_7_	
	Male (*n* = 22)	Female (*n* = 17)	Male (*n* = 22)	Female (*n* = 17)	Male (*n* = 22)	Female (*n* = 17)	Male (*n* = 22)	Female (*n* = 17)	Male (*n* = 22)	Female (*n* = 17)
a	18.1 ± 0.7	17.0 ± 1.1^∗^	18.7 ± 1.0	17.9 ± 1.1^∗^	18.9 ± 1.3	18.2 ± 1.0	20.5 ± 0.8	19.3 ± 1.1^∗^	22.2 ± 1.3	20.9 ± 1.0^∗^
b	19.2 ± 0.8	18.3 ± 0.8^∗^	20.0 ± 1.0	19.1 ± 0.7^∗^	20.3 ± 0.6	19.4 ± 0.6^∗^	22.2 ± 1.2	20.4 ± 1.1^∗^	23.4 ± 1.0	22.3 ± 1.3^∗^
c	20.5 ± 0.7	19.3 ± 0.6^∗^	21.1 ± 0.9	20.5 ± 0.5^∗^	21.6 ± 0.8	20.3 ± 1.0^∗^	23.0 ± 0.9	21.9 ± 1.1^∗^	24.7 ± 0.9	23.0 ± 0.7^∗^
d	18.5 ± 1.0	17.3 ± 1.2^∗^	19.1 ± 1.0	18.0 ± 0.7^∗^	19.5 ± 1.2	18.3 ± 1.0^∗^	21.2 ± 1.4	19.5 ± 1.2^∗^	22.3 ± 1.4	21.0 ± 1.1^∗^
e	19.8 ± 1.1	18.4 ± 0.8^∗^	20.7 ± 1.1	19.4 ± 1.0^∗^	20.9 ± 0.7	19.5 ± 1.3^∗^	22.4 ± 1.4	20.8 ± 1.0^∗^	24.0 ± 0.9	22.6 ± 1.2^∗^
f	20.8 ± 0.7	19.3 ± 1.1^∗^	21.4 ± 1.1	20.5 ± 0.9^∗^	21.8 ± 1.3	20.7 ± 0.9^∗^	23.1 ± 1.3	21.9 ± 0.5^∗^	25.0 ± 0.8	23.5 ± 0.9^∗^
g	20.2 ± 0.5	18.9 ± 1.1^∗^	20.3 ± 0.8	19.0 ± 0.8^∗^	21.1 ± 1.0	19.4 ± 1.0^∗^	22.4 ± 1.1	20.3 ± 0.9^∗^	23.8 ± 1.5	22.4 ± 0.8^∗^
h	21.5 ± 1.1	19.7 ± 0.9^∗^	21.7 ± 0.8	20.1 ± 1.2^∗^	22.4 ± 0.9	20.8 ± 0.5^∗^	23.8 ± 1.2	21.5 ± 0.9^∗^	25.1 ± 1.1	23.6 ± 1.4^∗^
i	22.4 ± 0.8	20.6 ± 1.2^∗^	23.1 ± 0.8	21.2 ± 1.0^∗^	23.5 ± 0.8	21.7 ± 1.1^∗^	24.9 ± 1.1	22.6 ± 0.8^∗^	26.2 ± 1.1	24.7 ± 0.7^∗^

Notes: ^∗^*P* < 0.05*vs*. male.

The article "Anatomical and Imaging Study on the Optimum Entry Point and Trajectory for Anterior Transpedicular Root Screw Placement into the Lower Cervical Spine" was published in 2022. Journal: Comput Math Methods Med.

**Table 2:** Comparison of horizontal angles of screws in different segments and regions (°).

	C_3_		C_4_		C_5_		C_6_		C_7_	
	Male (*n* = 22)	Female (*n* = 17)	Male (*n* = 22)	Female (*n* = 17)	Male (*n* = 22)	Female (*n* = 17)	Male (*n* = 22)	Female (*n* = 17)	Male (*n* = 22)	Female (*n* = 17)
a	45.4 ± 5.1	43.5 ± 2.8	45.2 ± 3.2	43.1 ± 3.5	44.0 ± 3.8	40.5 ± 2.4^∗^	43.4 ± 3.2	42.8 ± 3.3	45.7 ± 4.0	43.7 ± 4.1
b	41.1 ± 3.2	38.6 ± 2.8^∗^	39.4 ± 2.9	35.0 ± 3.4^∗^	36.4 ± 2.3	35.2 ± 3.8	36.4 ± 2.5	35.2 ± 3.0	38.5 ± 2.5	35.7 ± 4.2^∗^
c	34.1 ± 3.1	31.7 ± 2.6^∗^	33.2 ± 2.5	30.2 ± 3.8^∗^	34.0 ± 3.5	30.6 ± 3.4^∗^	33.0 ± 2.7	30.6 ± 2.3^∗^	33.1 ± 3.0	30.9 ± 4.0
d	46.2 ± 3.5	45.2 ± 2.9	44.1 ± 3.2	42.1 ± 2.6^∗^	44.1 ± 2.8	41.5 ± 4.0^∗^	43.5 ± 3.6	42.9 ± 3.8	44.7 ± 2.4	44.5 ± 3.7
e	41.5 ± 2.0	38.2 ± 4.1^∗^	40.3 ± 2.2	35.9 ± 3.9^∗^	36.2 ± 3.7	36.1 ± 2.9	35.9 ± 3.2	35.4 ± 4.1	37.4 ± 2.9	36.9 ± 3.2
f	36.4 ± 2.5	33.7 ± 3.5^∗^	34.5 ± 2.3	30.8 ± 3.7^∗^	33.4 ± 3.6	31.5 ± 3.6	31.6 ± 2.1	30.1 ± 2.8	33.8 ± 2.3	31.7 ± 3.4^∗^
g	44.2 ± 2.9	45.5 ± 2.4	47.1 ± 3.2	43.2 ± 3.8^∗^	45.8 ± 2.4	44.1 ± 2.1^∗^	44.8 ± 2.7	44.9 ± 3.3	46.2 ± 3.6	45.1 ± 4.2
h	41.2 ± 2.4	38.5 ± 3.9^∗^	40.8 ± 3.8	35.5 ± 2.4^∗^	39.3 ± 2.7	37.5 ± 2.2^∗^	38.6 ± 3.1	36.2 ± 2.5^∗^	38.3 ± 3.8	36.2 ± 4.2
i	36.8 ± 2.2	33.6 ± 2.9^∗^	35.2 ± 3.4	33.5 ± 1.9^∗^	34.4 ± 2.9	34.5 ± 3.2	33.8 ± 2.6	32.6 ± 3.4	34.2 ± 4.3	32.9 ± 3.4

Notes: ^∗^*P* < 0.05*vs*. male.

The article "Anatomical and Imaging Study on the Optimum Entry Point and Trajectory for Anterior Transpedicular Root Screw Placement into the Lower Cervical Spine" was published in 2022. Journal: Comput Math Methods Med.

**Table 3:** Comparison of sagittal angles of screws in different segments and zones (°).

	C_3_		C_4_		C_5_		C_6_		C_7_	
	Male (*n* = 22)	Female (*n* = 17)	Male (*n* = 22)	Female (*n* = 17)	Male (*n* = 22)	Female (*n* = 17)	Male (*n* = 22)	Female (*n* = 17)	Male (*n* = 22)	Female (*n* = 17)
a	86.2 ± 4.9	86.5 ± 5.2	86.5 ± 4.6	85.3 ± 4.2	93.2 ± 5.0	85.4 ± 5.7^∗^	92.1 ± 5.2	87.9 ± 4.9^∗^	86.7 ± 4.5	87.4 ± 4.9
b	85.6 ± 5.2	87.3 ± 4.8	93.2 ± 4.0	83.5 ± 4.3^∗^	95.6 ± 4.5	86.2 ± 4.3^∗^	94.5 ± 5.0	89.0 ± 5.7^∗^	89.3 ± 5.7	87.2 ± 3.9
c	86.2 ± 4.8	86.5 ± 5.0	92.7 ± 5.1	82.1 ± 4.1^∗^	97.2 ± 5.3	89.1 ± 4.2^∗^	91.8 ± 4.6	85.5 ± 3.6^∗^	86.4 ± 4.9	87.4 ± 4.2
d	104.2 ± 4.9	105.4 ± 5.1	106.7 ± 3.9	105.5 ± 4.1	110.4 ± 3.5	105.5 ± 3.8^∗^	109.2 ± 4.2	102.3 ± 3.7^∗^	104.3 ± 5.1	103.4 ± 4.0
e	106.7 ± 4.5	107.2 ± 5.3	107.5 ± 3.9	106.0 ± 4.4	113.4 ± 3.6	108.2 ± 4.3^∗^	111.3 ± 3.8	105.2 ± 2.9^∗^	107.5 ± 4.2	109.6 ± 4.8
f	101.3 ± 5.1	105.5 ± 3.8^∗^	108.1 ± 4.6	104.8 ± 4.5^∗^	112.0 ± 4.2	106.8 ± 3.8^∗^	110.6 ± 4.2	106.8 ± 3.1^∗^	109.4 ± 4.9	108.2 ± 4.5
g	121.4 ± 2.0	120.9 ± 5.2	123.7 ± 3.9	121.6 ± 4.2	124.9 ± 4.6	122.3 ± 4.9	124.5 ± 3.5	120.3 ± 4.6^∗^	116.2 ± 4.2	121.8 ± 3.8^∗^
h	122.4 ± 4.8	124.0 ± 4.1	125.4 ± 3.7	123.8 ± 4.0	125.4 ± 4.3	122.9 ± 5.6	123.4 ± 4.0	123.8 ± 3.8	119.0 ± 4.1	121.9 ± 4.0^∗^
i	122.6 ± 4.2	125.7 ± 5.3^∗^	125.2 ± 4.4	122.1 ± 4.7^∗^	128.3 ± 5.1	125.5 ± 5.0	122.2 ± 4.5	125.1 ± 5.2	123.8 ± 4.1	124.5 ± 3.9^∗^

Notes: ^∗^*P* < 0.05*vs*. male.

**Table 4:** Comparison of distance from the anterior midline of the VB to the P line at each segment (mm).

	C_3_	C_4_	C_5_	C_6_	C_7_
Male (*n* = 22)	8.2 ± 0.4	9.0 ± 0.5	9.3 ± 0.3	10.2 ± 0.3	14.1 ± 0.5
Female (*n* = 17)	7.5 ± 0.3	8.5 ± 0.3	9.1 ± 0.2	9.7 ± 0.4	12.8 ± 0.4
*t*	6.0184	3.6413	2.3685	4.4647	8.7624
*P*	<0.0001	0.0008	0.0232	<0.0001	<0.0001

## Data Availability

The labeled dataset used to support the findings of this study are available from the corresponding author upon request.
